The article "The design of tourism product CAD three-dimensional modeling system using VR technology" was retracted in 2024. Reasons: unreliable results or conclusions; concerns about the peer review.

# The design of tourism product CAD three-dimensional modeling system using VR technology

**DOI:** 10.1371/journal.pone.0244205

**Published:** 2020-12-28

**Authors:** Yilin Deng, Sang-Yun Han, Jianyi Li, Jinjin Rong, Wenyu Fan, Tiancong Sun

**Affiliations:** 1 College of Arts, Guilin University of Technology, Guilin, Guangxi, China; 2 College of Design and Media Entertainment, Hanseo University, Seosan-si, Chungcheongnam-do, Korea; 3 Guangxi Zhuang Autonomous Region Virtual Simulation Experimental Teaching Centre of Art and Design, Guilin, Guangxi, China; University College London, UNITED KINGDOM

## Abstract

In view of the high homogeneity of tourism products all over the country, an attempt is made to design virtual visit tourism products with cultural experience background, which can reflect the characteristics of culture + tourism in different scenic spots, so that tourists can deeply experience the local culture. Combined with computer aided design (CAD), the virtual three-dimensional (3D) modeling system of scenic spots is designed, and VR real scene visit interactive tourism products suitable for different scenic spots are designed. 360° VR panoramic display technology is used for 360° VR panoramic video shooting and visiting system display production of Elephant Trunk Hill park scenery. A total of 157 images are collected and 720 cloud panoramic interactive H5 tool is selected to produce a display system suitable for 360° VR panoramic display of scenic spots. Meanwhile, based on single view RGB-D image, the latest convolutional neural network (CNN) algorithm and point cloud processing algorithm are used to design the indoor 3D scene reconstruction algorithm based on semantic understanding. Experiments show that the pixel accuracy and mean intersection over union of the indoor scene layout segmentation network segmentation results are 89.5% and 60.9%, respectively, that is, it has high accuracy. The VR real scene visit interactive tourism product can make tourists have a more immersive sense of interaction and experience before, during and after the tour.

## Introduction

With the increasing level of China’s economic development, the composition of people’s daily life has also changed, and sightseeing and leisure has become a part of people’s life [1]. However, with the continuous development of tourism, tourism products are gradually homogenized. Tourists will feel that no matter where they go, they are all in the same scenic spot. Such a phenomenon needs to be improved and solved [2]. It is necessary to improve the personality of tourism products, and show the different characteristics and styles of different scenic spots, so that each scenic spot has its unique charm and attraction [3]. In view of the fierce competition in today’s tourism industry, it is necessary to combine the corresponding intelligent technology in tourism publicity to highlight the characteristics of local tourist scenic spots. Local customs, historical legends and other cultural experiences play a prominent role in distinguishing the homogeneity between scenic spots. The real world is three-dimensional (3D), and the tourism products with two-dimensional renderings cannot achieve a good display effect. The real world is also real, and ordinary 3D display cannot achieve good authenticity, and cannot let the audience completely immersed in it [4]. Therefore, landscape panoramic display based on virtual reality (VR) technology has become an important choice in front of the audience. Virtual tourism products can not only integrate the characteristics of different scenic spots into the 3D modeling system, but also pay more attention to the emotional pleasure and psychological experience of tourists during the tour, with the characteristics of immersion and interaction, so that tourists can better understand the characteristics of the scenic spot, and obtain a quite better tourism experience [5].

VR technology 3D space experience strengthens the "people-oriented" design principle [6]. In the early stage, tourism products are mainly scenic spots, that is, tourism publicity products; in the middle stage, they are the core content of tourism; in the later stage, they are extended tourism products, such as relevant supporting facilities and tourist souvenirs [7]. Although virtual tourism products cannot replace real tourism, they can be used as a kind of propaganda and supplement of real tourism, which can stimulate users’ interest and expectation of real tourism destination, and attract users to travel on the spot. VR technology used in tourism publicity will greatly improve the willingness of potential tourists to visit the nearby scenic spots [8].

This exploration is based on the characteristics of 360° VR panoramic roaming. The multi angle VR production materials are shot in the experimental scenic spot, and the 360° VR panoramic video display system is produced through the analysis of the main perspective; at the same time, the convolutional neural network (CNN) algorithm and point cloud processing algorithm are used to build the 3D model of the single view image captured by computer aided design (CAD). This exploration aims to design a tourist attraction publicity and guide system through VR technology and CAD 3D modeling system. This point-to-face combination can make the VR real scene visit interactive tourism products more authentic and experiential, and provide technical support for the scenic spot to attract tourists, promote characteristics and develop differentiated tourism.

## Method

### VR technology and tourism product design

VR technology enables users to interact with virtual environment with the help of relevant devices (VR head display, VR glasses, and mobile VR). It is a new technology combining computer graphics, human-computer interaction, multimedia and network technology [9]. 360° VR panoramic display technology can display all the sceneries in the vertical 180° and horizontal 360° in the scene comprehensively; users can browse and display from various perspectives, and can move in six directions: up, down, left, right, front, and back. If panoramic equipment is used for experience, it will further enhance the experience of human-computer interaction; panoramic display technology integrates advanced network technology and new media technology, which can transmit panoramic materials with high quality and high speed, and enhance the display effect in all directions [10].

Present VR technology products are closer and closer to people’s lives, the cost of using VR technology is lower and lower, and there are more and more opportunities to use them. VR technology has officially entered the market [11]. In the field of tourism, VR technology has been used and achieved good results. The VR studio of the Palace Museum not only meets the needs of tourists, but also achieves the purpose of displaying exhibits in the museum, and its security has been greatly improved [12]. At present, VR technology develops rapidly, and it has broad application prospects in many fields. For example, VR experience in tourist destinations, restoration of special perspectives and seasons, selection of hotel by VR experience, and digital virtual experience of VR museum are all application examples of VR technology [13].

The design of tourism products adopts the method of VR panoramic roaming and touch interaction. Compared with panoramic images and panoramic videos, the interactivity has been greatly improved. In addition to the basic 360° rotating viewing, panoramic roaming provides users with the opportunity to choose their own personality. It realizes the transformation from the previous experience mode of "seeing what is provided" to the brand-new experience mode of "seeing what they want to see", so as to meet the individual needs of user experience to the greatest extent. Even if there are many different needs in the development, according to these requirements, a variety of functional expansion can also be completed [14]. Fig 1 shows the system concept of VR real scene visit interactive tourism products.

**Fig 1:** Design of VR real scene tourism product system.

### Collection, analysis and display of multi angle shooting images

There are mainly three kinds of production methods of VR real scene visit interactive tourism product materials: field video shooting, two-dimensional image shooting and later 3D modeling. Among them, the frequency of field video shooting and post 3D production is relatively higher. The field shooting of panoramic display is generally to collect the image information of the environment to be displayed through the panoramic camera equipment. Panoramic images and panoramic video can be achieved through field shooting, and most of them need post-processing after shooting to export 360° panoramic video [15]. The production method of 3D modeling is mostly used in panoramic display system, which is also based on the real scene. The production process is mostly completed by the steps of preliminary planning, field investigation, design and display scheme, 3D modeling and model integration, and finally the interactive function is realized [16].

Different scenic spots have different geographical and cultural environment. In order to adapt to the panoramic video shooting link of each scenic spot to the maximum extent and reduce the difficulty of video and image data shooting in panoramic display, after analysis and research, the Insta360 ONE panoramic camera and Go Pro panoramic bracket are selected for shooting. Insta360 ONE panoramic camera has 1080P high definition real-time preview function, with 6*F2.4 fisheye lens, and can be used to take 12000 × 12000 ultra-high-resolution photos, which can meet the needs of this exploration. There are 8 positions in the Go Pro panoramic bracket, which can shoot seamless panoramic materials easily and quickly, and it is easy to operate in the later stage, which greatly saves time. The image of Go Pro panoramic bracket has good imaging effect and high definition. The panoramic image with good quality can be obtained by splicing Nuke and Cara VR plug-ins; considering the cost performance and production time, and the need to take panoramic images and panoramic videos at the same time, the How State super anti jitter technology in some mobile lens Insta360 ONE can play a key role in preventing the image from shaking.

In the process of multi angle video shooting in scenic spots, it is necessary to analyze the perspective area in each image to ensure the smooth switching of perspective in post-production. The 360° image range in panoramic display is divided into primary visual field, secondary visual field and blind visual field. The primary visual field is the front area that the user can directly see when watching, and the approximate angle range is 90°; the secondary visual field is the left and right side area, which can be seen by the residual light, and the approximate angle range is 70° respectively; the 130° behind is the blind visual field of the user’s whole landscape, and important images should be avoided as far as possible in the blind area of the user’s line of sight. Fig 2 shows the analysis area of tourists’ VR experience vision.

**Fig 2:** Analysis area of tourists’ VR experience vision.

After the creation of panoramic display is completed, in order to make users get better experience effect, panoramic display equipment is also essential. The existing panoramic display equipment mainly includes traditional screen and head mounted VR display equipment. In the VR real scene visit interactive tourism products experience, these two kinds of equipment are also taken. In the tourist experience center of the scenic area, the head mounted VR display device is used to experience VR real scenes visit interactive tourism products. It mainly includes three types of products: VR glasses for smart phones, VR all-in-one machine and VR devices on PC; after the tour of the scenic spot, if the tourists want to experience the VR real scene visit interactive tourism products again, they can scan the tickets of the scenic spot or the product two-dimensional code provided on other platforms of the scenic spot, enter the VR visiting system from the smartphone screen, and connect to the VR all-in-one device to experience.

Through the above analysis, according to the characteristics of different scenic spots, the interactive needs of tourists and the basic expression techniques of VR panoramic technology display, the multi angle shooting and display scheme of VR real scene visit interactive tourism products in scenic spots are determined as follows.

1. Panoramic camera is used to collect the panoramic image and panoramic video of the scenic spot, and the panoramic image roaming and panoramic video are used to display the scenic spot landscape.
2. For materials that have been shot, color matching, splicing, packaging and other work are carried out to complete the content of panoramic display.
3. The tickets and indicators of scenic spots with the two-dimensional code of VR real scene visit interactive tourism product experience are designed, so that users can scan the two-dimensional code on the tickets or indicators to see the VR panoramic roaming system of the actual scenic spots, and the tourist route is guided.

The domestic 720 cloud panoramic interactive H5 tool is selected as the panoramic image roaming creation tool. In cloud 720, multiple panoramic images can be inserted into panoramic image roaming, and various interactive effects such as logo, hotspot, sand table, mask, music, special effects, interpretation, guidance, and footprints can be inserted in panoramic roaming.

### Construction of 3D image of single view

The indoor objects in scenic spots are usually protected and maintained, so it is difficult to take full pictures from multiple angles. Therefore, it is very important to reconstruct CAD model with single view two-dimensional graphics. CAD 3D model reconstruction usually refers to the process of reconstructing the relative position of other indoor objects placed and decorated except the supporting plane. An attempt is made to complete the reconstruction of 3D model by matching the best model of indoor objects in scenic spots from the CAD model library published by authoritative organizations.

In different scenic spots, there are complex structures and many objects in the indoor scenic spots. In addition, the supporting planes such as ceiling, wall and floor and large indoor decorations make it relatively difficult to take multi angle image shooting under the close relationship between the two types of entities. The 3D scene composed of them is also quite complex, with great differences [17].

In order to meet the actual needs, a 3D reconstruction technology scheme based on semantic understanding to RGB-D indoor scene is adopted. Indoor scene layout estimation refers to the estimation of the relationship between the position and structure of the indoor support plane in the 3D scene according to the input indoor scene map. The scene layout estimation based on the depth information is incomplete, and the 3D model can only be reconstructed based on the Manhattan-world assumption [18]. CAD model reconstruction of indoor objects refers to the reconstruction process of other indoor objects except support plane. The method of finding the CAD model that best matches reconstruction target from the existing CAD model base is considered to replace the model reconstruction process. The premise of matching is to segment each reconstruction object from the scene one by one. It is necessary to combine the above two steps of reconstruction model to form a complete 3D indoor scene construction, and add color information to the model; finally, rendered images that can be viewed from any angle are output. Fig 3 shows the 3D image modeling system.

**Fig 3:** 3D image modeling system.

In conclusion, in order to improve the accuracy of 3D scene reconstruction under single view image, depth information of target scene is introduced. A complete scheme of indoor scene CAD model reconstruction using single view RGB-D image is proposed. CNN, point cloud data processing and other technologies are adopted. In this exploration, some evaluation indexes in computer vision and computer graphics are used for reference to evaluate and analyze the results. The experiments are carried out on the local RGB-D dataset and ShapeNet, a large-scale CAD model library provided by Stanford University. RGB-D dataset is a public dataset published by Computer Vision Lab of Technical University of Munich (TUM). The dataset is collected by Kinect, including depth image, RGB image, and ground truth data, which can be used for the system design here.

The following processing steps are adopted to realize the overall indoor 3D reconstruction technology scheme.

1. The RGB-D dataset is established and expanded. The input RGB-D image pairs are simply preprocessed, including equalization and restoration depth map.
2. Fully convolutional networks (FCN) is used to process the input RGB images, and the indoor scene layout is segmented by pixels.
3. The point cloud normal vector is estimated by depth image, and the indoor scene layout is estimated by combining the results in step (2).
4. Mask R-CNN network is used to detect and segment furniture entities in RGB images.
5. The detection results in step (4) are input into the self-coding neural network, and the CAD model rendering image with the highest similarity is matched in ShapeNet library.
6. The point cloud data in step (4) and the CAD model retrieved in step (5) are matched to complete the model positioning and pose correction.
7. The reconstruction results in step (3) and step (6) are combined to reconstruct the CAD model of the original scene, optimize the reconstruction model and output the rendering image.

For the RGB-D dataset involved in the method, the local dataset will be expanded and established with reference to the open RGB-D dataset. For the CAD model library, ShapeNet is directly used. The model library is provided by Stanford University. It contains more than 300,000 CAD models and is divided into 3135 common object categories. ShapeNet dataset provides consistent vertical and frontal correction for all models, and standardizes the model size to a unit length cube, so that all model data are aligned with the real physical world [19, 20].

In order to measure the proportion of various situations in pixel segmentation results, there are two commonly used evaluation indexes: pixel accuracy (PA) and mean intersection over union (mean IOU). In order to check the accuracy of defining the overlapped parts and boundaries between objects, Fig 4 is input into the system. The left circular area is the true value area, which is marked as A, and the right circular area is the prediction area, which is marked as B. The intersection of two shapes A and B is C, and C is the correct prediction area.

**Fig 4:** Inspection chart of 3D construction system.

The calculation equation of PA is as follows.

$$PA=\frac{\sum {}_{i}n_{ij}}{\sum {}_{i}t_{i}}$$ (1)

*n*_*ij*_ is the number of pixels with label *i* but predicted as tag *j*, and *t*_*i*_ *= ∑*_*j*_*n*_*ij*_ is the number of pixels labeled *i*.

The calculation equation of mean IOU (MI) is as follows.

$$MI=\frac{1}{n_{cl}}\sum_{i}\frac{n_{ii}}{t_{i}+\sum {}_{j}n_{ij}-n_{ii}}$$ (2)

*n*_*ij*_ and *t*_*i*_ are defined as above, and *n*_*cl*_ is the number of label categories.

CNN is used to extract semantic information from the target scene. Considering that the prior knowledge about the appearance and shape of interior decoration can be obtained from the rich CAD model base, by introducing large-scale CAD model library, the indoor layout is matched with the appropriate 3D model, and its position and posture are determined by using the point cloud information, so as to construct a complete VR panoramic tourism product.

## Results and discussion

### Panoramic VR display effect of multi angle shooting images

In this exploration, through the field shooting of Elephant Trunk Hill park, a total of 157 images are collected. Among them, 87 panoramas and 70 two-dimensional images are selected to show some classic scenes. In the panoramic roaming, the interactive experience is enriched by adding the images, texts, national commentators and lectures of historical and cultural stories. At the same time, in order to increase the experience effect of panoramic display and enhance the aesthetic feeling, the plane map of the Elephant Trunk Hill park is redrawn, and the maps that can have panoramic experience are marked and the conversion hotspot is added. Users can switch between the marked points in the scene or the scene selection method at the bottom of the interface to switch the scene. Fig 5a and 5b show the pages of VR scenic guide system in scenic spots.

**Fig 5:** **a.** Panoramic VR effect of scenic spots. **b.** Panoramic VR orientation display of scenic spots.

In addition, due to the 360° viewing angle of VR video, there is no change of scene in the design of panoramic video image splitting, so special attention should be paid to the problem of main view angle and the switching between panoramic images. Due to the large content of the panoramic image, it is necessary to leave enough viewing time for the viewer on each lens. In the actual design process, 8s viewing time is set for each lens. If the reservation time is short, tourists will have a serious sense of vertigo and discomfort on the screen content, which will affect the viewing experience of tourists.

### 3D modeling reconstruction effect of single view image

According to the method and equation introduced above, Table 1 shows all the results after calculation.

**Table 1:** Accuracy of FCN in judging overlapped pixels of objects.

	PA (%)	MI (%)
**Covered surface**	86.8	51.2
**Uncovered surface**	93.5	74.6
**Whole**	90.3	67.5

At the same time, the accuracy of judging overlapped pixels of the proposed method is compared with that of Hedau, Gupta, Ramalingam, Del Pero, Schwing, Mallya. Fig 6 shows the result. The classic semantic segmentation network FCN is used to segment indoor layout pixel by pixel. The results show that segmentation PA and mean IOU of FCN are 90.3% and 67.5%, respectively; meanwhile, the comparative analysis results show that the proposed method has a certain degree of improvement in judging and cutting overlapped objects than other algorithms. This method can match the two-dimensional images of scenic spots from the model library to the CAD model which has a high similarity with the observation results of indoor landscape reconstruction, so as to complete the design of VR panoramic model tourism products. In conclusion, the use of VR technology and CAD 3D modeling technology can enrich the effect of Elephant Trunk Hill park tour guide, make tourists get the experience of immersive tourism, and enrich the publicity means of the scenic spot. Based on the image effect of single view 3D modeling, the accuracy of overlapping pixels in this method is higher than that of Hedau, Gupta, Ramalingam, Del Pero, Schwing, and Mallya.

**Fig 6:** Comparison of PA of each method.

In addition, two eigenvalues, voxel Prec and voxel Recall are used to evaluate the completion of 3D model reconstruction, and the proportion of true value data from point cloud data is investigated. Table 2 shows the evaluation results of 3D model reconstruction.

**Table 2:** Evaluation of 3D model reconstruction effect.

Method	Data Set	voxel Prec	voxel Recall
**Gupta**	NYU Depth v2	0.912	0.925
**The proposed method**	NYU Depth v2	0.938	0.936
**The proposed method**	Text Data Set	0.942	0.928

The results show that in the NYU Depth v2 dataset, the voxel Prec and voxel Recall eigenvalues of Gupta method are 0.912 and 0.925, respectively, while those of the proposed method are finally 0.942 and 0.928. No matter on the NYU Depth v2 open dataset of New York University, or on the proposed dataset, the performance of 3D model reconstruction is better and the degree of completion is higher.

## Conclusion

Based on the development of VR technology, VR technology and CAD 3D modeling technology are combined to design VR real scene visit interactive tourism products for scenic spots. Through the VR panoramic display technology, the Elephant Trunk Hill park scenery is captured by VR panoramic video shooting and visiting system display production, a total of 157 images are collected. There are 87 panoramic images and 70 two-dimensional images. The domestic 720 cloud panoramic interactive H5 tool is selected to carry out systematic theoretical research and practical work, and a display scheme suitable for VR panoramic display of scenic spots is explored. According to the characteristics of different scenic spots, the display form of panoramic image roaming and panoramic video is determined, and the shooting, production and display media are analyzed and studied. At the same time, based on the single view RGB-D image and the prior knowledge of the shape of the target in the indoor scene, the large-scale CAD model library is introduced. The latest CNN algorithm and point cloud processing algorithm are used design an indoor 3D scene reconstruction algorithm based on semantic understanding, and the feasibility of the algorithm is verified on the local RGB-D dataset. Experimental results show that the PA and mean IOU of the segmentation results of the indoor scene layout segmentation network are 89.5% and 60.9%, respectively, which are consistent with the original scene. The reconstruction result combined with the normal vector of point cloud is consistent with the original scene.

In the way of VR panoramic video shooting and 3D reconstruction of indoor landscape two-dimensional image, a new display mode and technical mean for the research and development of scenic spot display are provided by using the frontier technology in the field of VR. Moreover, the panoramic display of scenic spots is shared by using mobile Internet technology. The design of VR real scene visit interactive tourism products provides tourists with a new way to visit, and also provides new publicity content and methods for different scenic spots. Based on this exploration, the number of VR images can be further increased, and the natural scenery and cultural characteristics of the scenic spot can be fully displayed.

## Supporting information

S1 Fig (VSDX)

S2 Fig (VSDX)

S3 Fig (VSDX)

S4 Fig (VSDX)

S5 Fig (JPG)

S6 Fig (OPJ)

S1 Data (XLSX)
